The article "Filters in 2D and 3D Cardiac SPECT Image Processing" was published in 2014. Journal: Cardiol Res Pract.

# Filters in 2D and 3D Cardiac SPECT Image Processing

**DOI:** 10.1155/2014/963264

**Published:** 2014-04-01

**Authors:** Maria Lyra, Agapi Ploussi, Maritina Rouchota, Stella Synefia

**Affiliations:** ^1^1st Department of Radiology, Faculty of Medicine, Aretaieion Hospital, University of Athens, 11528 Athens, Greece; ^2^2nd Department of Radiology, Faculty of Medicine, Aretaieion Hospital, University of Athens, 11528 Athens, Greece

## Abstract

Nuclear cardiac imaging is a noninvasive, sensitive method providing information on cardiac structure and physiology. Single photon emission tomography (SPECT) evaluates myocardial perfusion, viability, and function and is widely used in clinical routine. The quality of the tomographic image is a key for accurate diagnosis. Image filtering, a mathematical processing, compensates for loss of detail in an image while reducing image noise, and it can improve the image resolution and limit the degradation of the image. SPECT images are then reconstructed, either by filter back projection (FBP) analytical technique or iteratively, by algebraic methods. The aim of this study is to review filters in cardiac 2D, 3D, and 4D SPECT applications and how these affect the image quality mirroring the diagnostic accuracy of SPECT images. Several filters, including the Hanning, Butterworth, and Parzen filters, were evaluated in combination with the two reconstruction methods as well as with a specified MatLab program. Results showed that for both 3D and 4D cardiac SPECT the Butterworth filter, for different critical frequencies and orders, produced the best results. Between the two reconstruction methods, the iterative one might be more appropriate for cardiac SPECT, since it improves lesion detectability due to the significant improvement of image contrast.

## 1. Introduction

Cardiovascular disease (CVD) is a general term used to encompass various types of heart disease, including coronary heart disease (ischemic heart disease), pulmonary heart disease, stroke (cerebrovascular disease), diseases of arteries and other diseases of veins, heart failure, and rheumatic heart disease. CVD is the leading cause of death in the developed world accounting for approximately 17 million deaths per year. It is estimated that CVD is responsible for around 1 in every 3 deaths in men and 1 in every 5 deaths in women. CVD affects infant, children, and adults, both genders, and all ethnicities [1].

It has been observed that in many cases CVD events are connected to diseases such as chronic kidney disease (CKD) and metabolic syndrome (MetS) [2]. Such diseases may act as strong predictors of CVD, allowing an earlier diagnosis.

Nuclear imaging plays an important role and is considered a current standard in the diagnosis of CVD. Single photon emission tomography (SPECT) and positron emission tomography (PET) techniques evaluating myocardial perfusion, viability, and function are widely used in clinical routine [3].

The article "Filters in 2D and 3D Cardiac SPECT Image Processing" was published in 2014. Journal: Cardiol Res Pract.

The quality of the tomographic image is a key for the accurate diagnosis. Image filtering can greatly improve the image quality and yield information that otherwise could have been missed. There are several types of filters used in medical imaging and the choice of the appropriate filter in clinical practice is not an easy work [4].

Through cardiac SPECT myocardial perfusion defects as well as the overall coronary artery disease (CAD) can be detected. 3D surface images of the myocardium provide a relationship between the location and the degree of the stenosis in coronary arteries and the observed perfusion on the myocardial scintigraphy. The impact evolution of these stenoses can then be predicted and coronarography can be justified or avoided.

## 2. Basic Principles of Cardiac SPECT Imaging

### 2.1. Myocardium Data Acquisition

SPECT provides three-dimensional images that facilitate both a visual and a quantitative evaluation of the cardiac radionuclide distribution and of the surrounding tissues by removing superimposed activity from surrounding tissues [5].

The administrated radioisotope in the patient's body emits single gamma ray photons that are recorded through a gamma camera mounted on a gantry in numerous projections around the patient. Both contour and elliptical orbits can be used. The projection acquisition may be performed in three different ways: step-and-shoot, continuous, and continuous step-and-shoot. The method mostly used is the step-and-shoot method. For a given orbit, the camera stops at predefined angular positions and acquires a projection for predefined time durations. An arc of 180 degrees is usually covered, that is, 45 degrees right anterior oblique to left posterior oblique (RAO-LPO) [5]. Equal times are used to achieve the same count statistics.

Another parameter that greatly affects the image quality (sensitivity and resolution) is the choice of the collimator. This is determined mainly by the tracer activity. When ^201^Tl is being used a low-energy general purpose collimator is traditionally chosen. For ^99^Tc-labeled agents high resolution collimators are recommended, whereas for ^111^In and ^123^I—MIBG (metaiodobenzylguanidine) medium energy collimators are usually used [5].

Other important parameters that are to be taken into account during acquisition are the projection matrix size, the number of angles, and the time per view. For the projection matrix, a common rule of thumb is that at least three pixels should be used to image a structure for each full width at half maximum (FWHM) of the response profile. For the number of angles the time per view determines the statistical content of the projected image. The interrelationship of these parameters is quite complicated.

The article "Filters in 2D and 3D Cardiac SPECT Image Processing" was published in 2014. Journal: Cardiol Res Pract.

In most cardiac SPECT protocols, a 180° camera rotation with 64 × 64 matrix size is recommended [6]. The 2D projection-images are first corrected for nonuniformities and then mathematical algorithms are used to reconstruct 3D matrices of selected planes from the 2D projection data.

### 2.2. Myocardium Image Reconstruction Techniques

The purpose of reconstruction algorithms is to calculate an accurate 3D radioactivity distribution from the acquired projections. There are two methods to reconstruct SPECT images, either by filter back projection (FBP) analytical technique or iteratively, by algebraic methods.

#### 2.2.1. Filtered Back Projection Method (FBP)

Filtered back projection is an analytical method that is still the most widely used in clinical SPECT because of its simplicity, speed, and computational efficiency. FBP consists of two steps: filtering of data and back projection of the filtered data [7].

In 2D acquisition, each row of projections represents the sum of all counts along a straight line through the depth of the object being imaged. Back projection technique redistributes the number of counts at each particular point back along a line from which they were originally detected. This process is repeated for all pixels and all angles. A limited number of projection sets can result in the formation of the star artifact and in blurring of the image. To eliminate this problem, the projections are filtered before being back projected onto the image matrix. It has to be noticed that the back projection process has taken place in spatial domain while data filtration is done in the frequency domain. While the analytic approaches typically result in fast reconstruction algorithms, accuracy of the reconstructed images is limited by the approximations in the line-integral model on which the reconstruction formulae are based [8]. Cardiac SPECT reconstruction process may obtain attenuation corrections approximately, using a postprocessing step [9]. Some reconstruction algorithms apply approximation formulas to the projection data for attenuation correction. Lee-Tzuu [9] applied a simple, effective two-step procedure to the uncorrected image. For two-dimensional (2D) SPECT with parallel or fan beam collimators, 2D filtered back projection (FBP) algorithms are routinely used for myocardium SPECT reconstruction.

The article "Filters in 2D and 3D Cardiac SPECT Image Processing" was published in 2014. Journal: Cardiol Res Pract.

#### 2.2.2. Iterative Reconstruction Method

Iterative reconstruction starts with an initial estimate of the image [7]. Most of the times, the initial estimate is very simple, for example, a uniform activity distribution. Then a set of projection data is estimated from the initial estimate using a mathematical process called forward projection. The resulting projections are compared with the recorded projections and the differences between the two are used to update the estimated image. The iterative process is repeated until the differences between the calculated and measured data are smaller than a specified preselected value.

Data from SPECT systems using parallel, fan beam, and cone beam collimators can be modelled as sets of line integrals of the tracer density along the collimation directions. Consequently, SPECT images can be reconstructed using analytic inversion methods that are based on the relationship between a function and its line integrals.

For 3D SPECT, the iterative reconstruction methods include algebraic methods like the algebraic reconstruction technique (ART) and statistical algorithms like maximum likelihood expectation maximization (ML-EM) or ordered subsets expectation maximization (OS-EM) [10]. The ML-EM algorithm is a general approach to solving maximum likelihood problems through the introduction of a set of data which, if observed, would make the ML problem readily solvable. The algorithm then iterates between computing the mean of the complete data, given the observed data and the current estimate of the image, and maximizing the probability of the complete data over the image space. In the ordered subsets EM (OS-EM) method the full set of views is divided into subsets and the EM algorithm applied sequentially to each of these data sets in turn. This produces remarkable improvements in the initial convergence rate compared to ML-EM [8].

### 2.3. Image Processing in 3D and 4D Cardiac SPECT

After the planar images have been obtained for several projection angles, a 3D reconstruction can be performed using different methods and the appropriate filters. The first method is by using a type of commercially available software for SPECT imaging. Such software with different filters is discussed in Section 5.1. Another method is by using a specified programming code. Such a MatLab code is tested in Section 5.2, again for multiple filters. When a spatiotemporal approach is of need, electrocardiogram- (ECG-) gated SPECT can be performed. In ECG-gated SPECT, data from specific parts of the cardiac cycle can be isolated. This method is further explained in Section 6.

### 2.4. Image Filtering in Cardiac SPECT

Different filter types in SPECT imaging can produce different optimal results in processed images, such as star artifact reduction, noise suppression, or signal enhancement and restoration [4]. The choice of filter for a given image processing task is generally a compromise between the extent of noise reduction, fine detail suppression, and contrast enhancement, as well as the spatial frequency pattern of the image data of interest.

The article "Filters in 2D and 3D Cardiac SPECT Image Processing" was published in 2014. Journal: Cardiol Res Pract.

Filters that are commonly used on SPECT imaging are the Ramp filter, a high pass filter eliminating the star artifact and blurring, the Hanning filter, a low pass smoothing filter, the Hamming filter, also a low pass smoothing filter having a different amplitude at the cutoff frequency, the Butterworth filter, which both smoothers noise and preserves the image resolution, the Parzen filter, the most smoothing low pass filter, and the Shepp-Logan filter, which is the least smoothing but has the highest resolution [4]. Two enhancement filters also used in cardiac SPECT are the Metz filter, a function of modulation transfer function and the Wiener filter, which is based on the signal-to-noise ratio of the specific image.

The filters mostly used in cardiac SPECT imaging are presented with a greater detail in the next paragraphs. A more extensive presentation of all the mentioned filters can be found in “Filtering in SPECT Image Reconstruction” [11].

#### 2.4.1. Ramp Filter

The Ramp filter is the most widely used high pass filter, as it does not permit low frequencies that cause blurring to appear in the image. In frequency domain its mathematical function is given by

(1) $$\begin{array}{c} H_{R}\left(k_{x},k_{y}\right)=k=\sqrt{k_{x}^{2}+k_{y}^{2}}, \end{array}$$

where *k*_*x*_,  *k*_*y*_ are the spatial frequencies.

The Ramp is a compensatory filter as it eliminates the star artifact resulting from simple back projection. Because the blurring only appears in the transaxial plane, the filter is only applied in that plane [12]. The filter is linearly proportional to the spatial frequency. As a high pass filter the Ramp filter has the severe disadvantage of amplifying the statistical noise present in the measured counts. In order to reduce the amplification of high frequencies the Ramp filter is always combined with a low pass filter.

#### 2.4.2. Butterworth Filter

Butterworth filter is the filter mostly used in nuclear medicine. The Butterworth filter is a low pass filter. It is characterized by two parameters: the critical frequency, which is the point at which the filter starts its roll-off to zero and the order or power [13]. As it is mentioned earlier the order changes the slope of the filter. Because of this ability to change not only the critical frequency but also the steepness of the roll-off, the Butterworth filter can both smoothen noise and preserve the image resolution. A Butterworth filter in spatial domain is described by the following equation:

(2) $$\begin{array}{c} B\left(f\right)=\frac{1}{1+{\left(f/f_{c}\right)}^{2n}}, \end{array}$$

where *f* is the spatial frequency domain, *f*_*c*_ is the critical frequency, and *n* is the order of the filter.

The article "Filters in 2D and 3D Cardiac SPECT Image Processing" was published in 2014. Journal: Cardiol Res Pract.

Filtration is usually applied to projection images before reconstruction, but effect of filtration is shown on reconstructed transaxial images [6]. Because Butterworth filters are low pass filters, their application results in smoother images than with no filtering application.

Lower critical frequencies correspond to increased smoothing, with optimal value depending on specific radioisotope and protocol used. Power factor of a filter equals (by definition) twice its order, and all frequencies are expressed in cycles per centimeter rather than cycles per pixel.

The selection of the cutoff frequency is important to reduce noise and preserve the image details. The effect of Butterworth filter of various cutoff frequencies with order *n* = 5 (power 10) in a myocardial SPECT study, reconstructed by filtered back projection (FBP), is shown in Figure 1.

#### 2.4.3. Hanning Filter

The Hanning (or Hann) filter is a relatively simple low pass filter, which is described by one parameter, the cutoff frequency [14]. The Hanning filter is defined in the frequency domain as follows:

(3) $$\begin{array}{c} H\left(f\right)=\{\begin{array}{cc} 0.5+0.5\cos\left(\frac{\pi f}{f_{m}}\right), & 0\leq \left|f\right|\leq f_{m}\\ 0, & \text{otherwise}, \end{array} \end{array}$$

where *f* are the spatial frequencies of the image and  *f*_*m*_is the cutoff frequency. The Hanning filter is very effective in reducing image noise because it reaches zero very quickly. However, it does not preserve edges. The effect of varying cutoff frequencies for the Hanning filter for FBP reconstruction is shown in Figure 2.

#### 2.4.4. Parzen Filter

The Parzen filter is another example of a low pass filter and is defined in the frequency domain as follows [14]:

(4) $$\begin{array}{c} \left|f\right|-6\left|f\right|{\left(\frac{\left|f\right|}{f_{m}}\right)}^{2}\times \left(1-\frac{\left|f\right|}{f_{m}}\right)\;\;\left(\left|f\right|≺\frac{f_{m}}{2}\right),\\ P\left(f\right)=\{\begin{array}{cc} 2\left|f\right|{\left(1-\frac{\left|f\right|}{f_{m}}\right)}^{3}, & \left(\frac{f_{m}}{2}≺\left|f\right|≺f_{m}\right)\\ 0, & \left(\left|f\right|\geq f_{m}\right), \end{array} \end{array}$$

where *f* are the spatial frequencies of the image and  *f*_*m*_  is the cutoff frequency.

The article "Filters in 2D and 3D Cardiac SPECT Image Processing" was published in 2014. Journal: Cardiol Res Pract.

The Parzen filter is the most smoothing filter; it not only eliminates high frequency noise but it also degrades the image resolution [4].

#### 2.4.5. Metz Filter

The Metz filter is a function of modulation transfer function (MTF) and it is based on the measured MTF of the gamma camera system. The MTF describes how the system handles or degrades the frequencies. The Metz restoration filter is defined in the frequency domain as follows [19]:

(5) $$\begin{array}{c} M\left(f\right)=\text{MTF}{\left(f\right)}^{-1}\left[1-{\left(1-\text{MTF}{\left(f\right)}^{2}\right)}^{x}\right], \end{array}$$

where *f* is the spatial domain and *x* is a parameter that controls the extent to which the inverse filter is followed before the low pass filter rolls off to zero.

Equation (5) is the product of the inverse filter (first term) and a low pass filter (second term).

The Metz filter is count-dependent.

#### 2.4.6. Wiener Filter

The Wiener filter is based on the signal-to-noise ratio (SNR) of a specific image. The one-dimensional frequency domain form of the Wiener filter is defined as follows [20]:

(6) $$\begin{array}{c} W\left(f\right)={\text{MTF}}^{-1}\times \frac{{\text{MTF}}^{2}}{\left({\text{MTF}}^{2}+N/O\right)}, \end{array}$$

where MTF is the modulation transfer function of the imaging system, *N* is the noise power spectrum, and *O* is the object power spectrum. As with the Metz filter, the Wiener is the product of the inverse filter (which shows the resolution recovery) and the low pass filter (which shows the noise suppression). In order to apply the Wiener filter it is necessary to know a priori the MTF, the power spectrum of the object, and the power spectrum of the noise. It has to be noticed that is impossible to know exactly the MTF or the SNR in any image. As a result the mathematical models used to optimize both Metz and Wiener filters are uncertain [4].

#### 2.4.7. Cardiac SPECT Filter Dependence

Gamma camera systems offer a wide choice of filters in cardiac SPECT as well as in many types of examinations. The filter choice depends on several parameters [4, 21]:

- the energy of the isotope, the number of counts, and the activity administration;
- the statistical noise and the background noise level;
- the type of the organ being imaged;
- the kind of information we want to obtain from the images;
- the collimator that is used.

The choice of the filter must ensure the best compromise between the noise reduction and the resolution in the image.

## 3. A Comparison of Various Filters in Cardiac SPECT: Studies on Phantoms

Myocardial SPECT is a well-established, noninvasive technique to detect flow-limiting coronary artery disease during stress and rest conditions. Comparison of the myocardial distribution of radiopharmaceutical after stress and at rest provides information on myocardial viability, inducible perfusion abnormalities, regional myocardial motion, and thickening. In cardiac SPECT, the most commonly used radiotracers are thallium-201 (^201^Tl) and technetium-99m (^99m^Tc) labeled agents such as sestamibi and tetrafosmin. According to the literature, the sensitivity, specificity, and accuracy of cardiac SPECT varies from 71% to 98%, 33% to 89%, and 72% to 95%, respectively [22, 23].

The article "Filters in 2D and 3D Cardiac SPECT Image Processing" was published in 2014. Journal: Cardiol Res Pract.

The quality of the myocardium SPECT images is degraded by several factors. The most important factors affecting image quality of myocardial perfusion SPECT are the statistical fluctuation in photon detection, the attenuation of photons through the tissues, and the scatter radiation [24]. Especially, nuclear cardiology images, because of their relatively low counts statistics (breast attenuation, obesity patients), tend to have greater amount of image noise [25]. Image filtering is necessary to compensate these effects and therefore to improve image quality.

In order to test and improve the image quality in SPECT specially constructed phantoms are used for measurements. An example of such a phantom is the PET/SPECT performance phantom, designed and developed by Carlson and Colvin [26], Fluke Biomedical, Nuclear Associates (Figure 3). The effect of implementing different filters on the hot region of Carlson phantom SPECT image was tested in order to evaluate the perceived image quality of the hot region and also its detectability, as far as filters are concerned. The findings showed that the more accurate locations of radionuclide distribution were produced when using the Ram-Lak and Shepp-Logan filters with cutoff frequency of 0.4 [15].

A cardiac insert (Figure 3(d)) may be used with the Carlson phantom to mimic the human heart for myocardial perfusion study. The “heart” is approximately 8 cm in diameter and has a 1.5 cm thick hollow “wall,” which may be filled with a solution containing ^201^Tl or ^99m^Tc. The insert is placed within the source tank which could be filled with radioactive background solution [26]. Evaluation of cardiac ECT data acquisition and reconstruction methods can be performed as well as a quantitative evaluation of nonuniform attenuation and scatter compensation methods. Reconstruction of heart insert images helps in standardization.

Another three-dimensional simulator was created to meet the imaging needs of general and cardiac nuclear imaging departments by Medical Designs, Inc. (MDI). The SNMMI 2012 cardiac SPECT phantom simulator makes possible for myocardial perfusion studies to be performed and for areas of perfusion abnormality to be quantified. Findings can then be evaluated as far as their diagnostic and prognostic significance is concerned [16]. One can use it to perform both visual and semiquantitative evaluation of the images. A picture of SNMMI cardiac phantom is shown below (Figure 4).

The article "Filters in 2D and 3D Cardiac SPECT Image Processing" was published in 2014. Journal: Cardiol Res Pract.

The standardization of image processing confines the filter types for myocardium SPECT imaging to certain filters. Moreover, only specific values of cutoff frequency and order or power are selected to optimize image processing time and clinical results.

Takavar et al. [27] studied the determination of the optimum filter in ^99m^Tc myocardial SPECT using a phantom that simulates the heart left ventricle. Filters such as Parzen, Hanning, Hamming, and Butterworth and a combination of their characteristic parameters were applied on the phantom images. To choose the optimum filter for quantitative analysis contrast, signal-to-noise ratio (SNR) and defect size criteria were analyzed. In each of these criteria were given a number from 1 to 20, 1 for the worst and 20 for the best contrast and SNR, while 1 for the largest defect size and 20 for the smallest. For every filter, the final criterion resulted from the total sum of the marks of the previous parameters. The study showed that Parzen filter is inappropriate for heart study. The cutoff frequency of 0.325 Nq and 0.5 Nq gave the best overall result for Hanning and Hamming filters, respectively. For Butterworth filter order 11 and cutoff 0.45 Nq gave the best image quality and size accuracy.

A determination of the appropriate filter for myocardial SPECT was conducted by Salihin and Zakaria [14]. In this study a cardiac phantom was filled with 4.0 *μ*Ci/mL (0.148 MBq/mL) ^99m^Tc solution. The filters functions evaluated in this study included Butterworth, Hamming, Hanning, and Parzen filters. From these filters, 272 combinations of filter parameters were selected and applied to the projection data. For the determination of the best filter Tanavar et al. [27] method was applied [20]. The study suggested that Butterworth filter succeeds the best compromise between SNR and detail in the image while Parzen filter produced the best accurate size.

The same group [28] has investigated the relationship between the optimum cutoff frequency for Butterworth filter and lung-heart ratio in ^99m^Tc myocardial SPECT. For the study a cardiac phantom was used and the optimum cutoff frequency and order of Butterworth filter were determined using Takavar et al. method [27]. A linear relationship between cutoff frequency and lung-heart ratio had been found which shows that the lung-heart ratio of each patient must be taken into account in order to choose the optimum cutoff frequency for Butterworth filter.

The article "Filters in 2D and 3D Cardiac SPECT Image Processing" was published in 2014. Journal: Cardiol Res Pract.

Links et al. [20] examined the effect of Wiener filter in myocardial perfusion with ^201^Tl SPECT. The study was done in 19 dogs and showed that Wiener filter improves the quantization of regional myocardial perfusion defects.

In a myocardial perfusion study with ^99m^Tc sestamibi, the investigators explore the effect of different filters on the contrast of the defected location. Calculations showed that maximum contrast between normal and defected myocardium could be obtained using the Metz (FWHM 3.5–4.5 pixel, orders of 8–9.5), Wiener (FWHMs 3.5–4), Butterworth (cutoffs 0.3–0.5, orders 3–9) and Hanning (cutoffs 0.43–0.5) [29].

## 4. IR versus FBP in Cardiac SPECT

Iterative reconstruction (IR) algorithms allow accurate modelling of statistical fluctuation (noise), produce accurate images without streak artifacts as FBP, and promise noise suppression and improved resolution [30].

The most commonly used IR method in SPECT studies is ordered-subset expectation maximization (OSEM). Myocardial perfusion SPECT images reconstructed with OSEM IR algorithm have a superior quality than those processed with FBP. Perfusion defects, anatomic variants, and the right ventricular myocardium are better visualized with OSEM. Likewise, image contrast is improved, thereby better defining the left ventricular endocardial borders. The effect of OSEM on image quality improvement is more intense in lower count density studies [31].

Hatton et al. [32], in myocardial perfusion SPECT study, show that OSEM technique demonstrates fewer artifacts and improves tolerance when projections are missing. However, OSEM seems to be less tolerant in motion artifacts than FBP [33]. Won et al. [34], in 2008, studied the impact of IR on myocardial perfusion imaging in 6 patients. The results demonstrate that there was no statistically significant difference in the accuracy of myocardial perfusion interpretation between FBP and IR but there were statistically significant differences in functional results.

A stress perfusion imaging study, reconstructed both by FBP and by OSEM algorithm, using the Butterworth filter, is shown in Figure 5. It is believed that in such a case diagnostic information might be easier to obtain through the OSEM algorithm. This is because corrections for image degrading effects, such as attenuation, scatter, and resolution degradation, as well as corrections for partial volume effects and missing data, are quite straightforward to be included in the resulting image through iterative techniques [35].

## 5. Reconstruction and Processing of 3D Cardiac SPECT Images

The 3-dimensional (3D) description of an organ and the information of an organ's surface can be obtained from a sequence of 2D slices reconstructed from projections to form a volume image. Volume visualization obtains volumetric signs useful in diagnosis, in a more familiar and realistic way. Filtering, thresholding, and gradient are necessary tools in the production of diagnostic 3D images [36].

The article "Filters in 2D and 3D Cardiac SPECT Image Processing" was published in 2014. Journal: Cardiol Res Pract.

Cardiac SPECT provides information with respect to the detection of myocardial perfusion defects, the assessment of the pattern of defect reversibility, and the overall detection of coronary artery disease (CAD). There is a relationship between the location and the degree of the stenosis in coronary arteries and the observed perfusion on the myocardial scintigraphy, using data of 3D surface images of myocardium. This allows us to predict the impact of evolution of these stenoses to justify a coronarography or to avoid it.

### 5.1. 3-Dimensional Software: Filter Application

Seret and Forthomme [37] have studied types of commercial software for SPECT image processing. It was also observed that there were 2 definitions of the Butterworth filter. For a fixed order and a fixed cutoff frequency, one definition led to a less smoothing filter, which resulted in higher noise levels and smaller FWHMs. However, differences in the FWHM were translated to differences in contrast only when they exceeded 0.5 mm for the hot rods and 1 mm for the cold rods of the used phantom. When considering the FWHM and noise level, more noticeable differences between the workstations were observed for OSEM reconstruction.

All of the software types used in the study [37] behaved as expected: lowering the filter cutoff frequency in FBP resulted in larger FWHMs and in lower noise levels and reduced contrast; increasing the product number of subsets times the number of iterations in OSEM resulted in improved contrast and higher noise levels.

Nowadays, in many cases myocardium diagnosis is relied on 3D surface shaded images. 3D data obtained at stress and at rest of the LV myocardium, respectively, are analysed and the deformation of both images is evaluated, qualitatively and quantitatively.

3D data reconstructed by IR were obtained by the G.E. Volumetrix software in the G.E. Xeleris processing system at stress and rest MPI studies (Figure 6). Butterworth Filter (cutoff frequency 0.4 cm^−1^, power 10) was used in both reconstructions. Chang attenuation correction was applied (coefficient = 0.1). These data were then used to evaluate the left ventricle deformation in both stress and rest 3D surface image series. If a significant difference is obtained in rest and stress 3D data perfusion, the location and the impact of the pathology of left ventricle myocardium are recognized.

3D shaded surface display of a patient stress and rest perfusion angular images (Figure 7) can be reconstructed by FBP or OSEM algorithm and improved, usually, by Butterworth or Hanning filter. 3D reconstruction in studies by Tc99m tetrofosmin may show normal (or abnormal) myocardium perfusion, in apex, base, and walls of myocardium. Transaxial slices are used to be reconstructed and the created 3D volume images are displayed. Through base we recognize the cavity of LV.

The article "Filters in 2D and 3D Cardiac SPECT Image Processing" was published in 2014. Journal: Cardiol Res Pract.

### 5.2. 3-Dimensional Reconstruction by MatLab: Filters Application

3D reconstruction was also performed using a specified MatLab code, in order to evaluate the different filters used (Figure 10) and also to compare myocardium volume at rest and at stress (Figure 11). In MatLab, volume visualization can be achieved by constructing a 3D surface plot which uses the pixel identities for (*x*, *y*) axes and the pixel value is transformed into surface plot height and, consequently, colour. Apart from that, 3D voxel images can be constructed; SPECT projections are acquired; isocontours are depicted on them including a number of voxels, and finally all of them can be added in order to create the desirable volume image [17]. The method is illustrated in Figures 8 and 9 for rest and stress conditions, respectively.

The volume rendered by MatLab is slow enough but similar to other codes' volume renderings.

The volume rendering used in 3D myocardium used zoom, angles of 5.6 degrees and a focal length in pixels depending on the organs' size. The size of the reprojection is the same as the main size of input image.

## 6. 4D Gated SPECT Imaging

In some cases SPECT imaging can be gated to the cardiac electrocardiogram signal, allowing data from specific parts of the cardiac cycle to be isolated and providing a spatiotemporal approach (4D). It also allows a combined evaluation of both myocardial perfusion and left ventricular (LV) function in one study, which can provide additional information that perfusion imaging cannot provide alone. An example of such a case are patients suffering from a 3-vessel coronary disease, where gated SPECT has been noted to yield significantly more abnormal segments than perfusion does alone [38].

As in a regular SPECT acquisition, a *γ*-camera registers photons emitted from the object at multiple projection angles, along an arc of usually 180 degrees. At each projection, instead of one static image, several dynamic images are acquired, spanning the length of the cardiac cycle, at equal intervals. The cardiac cycle is marked within the R-R interval, which corresponds to the end-diastole, and is divided in 8-16 equal frames. For each frame, image data are acquired over multiple cardiac cycles and stored. All data for a specific frame are then added together to form an image representing a specific phase of the cardiac cycle. If temporal frames are added together the resulting set of images is equivalent to a standard set of ungated perfusion images.

The article "Filters in 2D and 3D Cardiac SPECT Image Processing" was published in 2014. Journal: Cardiol Res Pract.

During reconstruction in gated SPECT a significant level of smoothing is required, in comparison to ungated or summed projection data, because of the relatively poor counts [39]. This is done by using appropriate filters. Several studies have been made to establish the most appropriate filters for this purpose.

In a ^201^Tl gated SPECT study, concerning patients with major myocardial infarction [40], a Butterworth filter of order 5, with six cutoff frequencies (0.13, 0.15, 0.20, 0.25, 0.30, and 0.35 cycle/pixel), was successively tested. The report showed that filtering affects end diastolic volume (EDV), end systolic volume (ESV), and left ventricular ejection fraction (LVEF). Marie et al. [41] suggested that the best results for cardiac gated SPECT image reconstruction with ^201^Tl were achieved using a Butterworth filter with an order of 5 and cutoff frequency 0.30 cycles/pixel.

In 2005 [42], the differences produced by change of reconstruction filter in calculations of left-ventricular end diastolic volume (EDV), end systolic volume (ESV), stroke volume (SV), and ejection fraction (LVEF) from ^99m^Tc-sestamibi myocardial gated SPECT studies have been investigated. Butterworth order 4, cutoff frequency 0.25 cycles /pixel and Metz order 8, full-width half maximum 4.0 mm were applied and compared. With the Metz filter rather than the Butterworth filter left-ventricular EDV and ESV were significantly larger, and the LVEF and SV were not significantly changed. The results were consistent to previous similar studies [40, 43].

## 7. Discussion

The SPECT filters can greatly affect the quality of clinical images. Proper filter selection and adequate smoothing helps the physician in results' interpretation and accurate diagnosis.

Several studies on phantoms with respect to the most appropriate filter for cardiac SPECT have been considered. The studies showed that for the 3D SPECT reconstruction Butterworth filter succeeds the best compromise between SNR and detail in the image, while Parzen filter produces the best accurate size [20]. Maximum contrast between normal and defected myocardium could be obtained using the Metz (FWHM 3.5–4.5 pixel, orders of 8–9.5), Wiener (FWHMs 3.5–4), Butterworth (cutoffs 0.3–0.5, orders 3–9), and Hanning (cutoffs 0.43–0.5) filters [29]. The cutoff frequency of 0.325 of  Nq gave the best overall result for the Hanning filter, whereas for the Butterworth filter, order 11 and cut off of 0.45 Nq gave the best image quality and size accuracy [27].

The article "Filters in 2D and 3D Cardiac SPECT Image Processing" was published in 2014. Journal: Cardiol Res Pract.

For the 4D ECG-gated SPECT reconstruction, best results were obtained using a Butterworth filter with an order of 5 and cutoff frequency of 0.30 cycles/pixel [41].

As far as the reconstruction technique is concerned, using 3D OSEM with suitable AC may improve lesion detectability due to the significant improvement of image contrast [35]. 3D iterative reconstruction algorithms are likely to replace the FBP technique for many SPECT clinical applications.

When a specified 3D reconstruction MatLab code was used to compare both two chosen filters (Butterworth and Hann) and myocardium volume at rest and at stress, accurate diagnostic images were produced.

It is expected that further significant improvement in image quality will be attained, which, in turn, will increase the confidence of image interpretation. The development of algorithms for analysis of myocardial 3D images may allow better evaluation of small and nontransmural myocardial defects. For the diagnosis and treatment of heart diseases, the accurate visualisation of the spatial heart shape, 3D volume of the LV, and the heart wall perfusion plays a crucial role. Surface shading is a valuable tool for determining the presence, extent and location of CAD.

Further developments in cardiac diagnosis include a new promising tool, computational cardiology. The functions of the diseased heart and the probable new techniques in diagnosis and treatment can be studied using state-of-the-art whole-heart models of electrophysiology and electromechanics. A characteristic example of implementing such a model is ventricular modelling, where important aspects of arrhythmias, including dynamic characteristics of ventricular fibrillation can be revealed. Performing patient-specific computer simulations of the function of the diseased heart for either diagnostic or treatment purposes could be an exciting new implementation of computational cardiology [44].

## Figures and Tables

**Figure 1:** The effect of varying cutoff frequencies of Butterworth filter of order 5 (power factor = 10 for all critical frequencies) with FBP. First column shows myocardial slices and second column shows Butterworth equation curves for various cutoff frequencies (0.2, 0.3, 0.5, and 0.8) in cycles/cm (minimum value 0.0 and maximum value 2.0).

**Figure 2:** The effect of varying cutoff frequencies of Hanning filter with FBP. First column shows myocardial slices and second column shows Hanning equation curves for various cutoff frequencies (0.5, 0.9, 1.2, and 1.6) in cycles/cm (minimum value 0.0 and maximum value 2.0).

The article "Filters in 2D and 3D Cardiac SPECT Image Processing" was published in 2014. Journal: Cardiol Res Pract.

**Figure 3:** (a) The Carlson phantom showing the individual inserts for resolution and contrast evaluation, (b) the phantom assembled, showing all inserts, including hot and cold regions, (c) schematic diagrams of the pairs holes as hot regions and drawn line profiles for evaluation of hot regions. (a)–(c) obtained from citation [15]. (d) Cardiac insert with solid/fillable defect set (Model ECT/CAR/I).

**Figure 4:** The SNMMI 2012 Cardiac SPECT phantom simulator showing the myocardium insert, manufacturedby Medical Designs, Inc. (MDI). Figure is obtained from citation [16].

**Figure 5:** Comparison of vertical, horizontal, and short axis slices of a stress perfusion imaging study reconstructed by FBP (a) and by OSEM (b) algorithm, using the Butterworth filter (cutoff frequency: 0.3 cm^−1^ and power 10) as a processing filter. Data acquired by GE Starcam 4000 and reconstructed in Radiation Physics Unit, University Aretaieion Hospital, Athens, Greece, 2013.

**Figure 6:** 3D reconstruction at stress (a) and rest (b), by OSEM iterative reconstruction (10 subsets), Butterworth filter (cutoff 0.4 Hz, power 10, Chang AC coefficient 0.1) obtained by the GE. Volumetrix software (GE. Xeleris-2 processing system). The colour scale indicates a high perfusion in white and red regions and a lower perfusion in the other regions. Defected areas are seen on the above image with a darker colour. A perfusion recovery of the defects on the rest images is observed. Data acquired by GE Starcam 4000 and reconstructed in Radiation Physics Unit, University Aretaieio hospital, Athens, Greece, 2013.

**Figure 7:** Stress (a) and at rest (b) 3D surface angular images of female myocardium. Small defect at posterior-basal wall at stress is improved, almost completely, at rest (2% rest defect); threshold value 50% of maximum. OSEM iterative reconstruction. Defect lesion under stress is recovered in rest condition (seen on the first structure in both above and below image).

**Figure 8:** Isocontour surfaces for threshold value determination, in rest [17]. Images obtained in Radiation Physics Unit, University Aretaieio hospital, Athens, Greece, 2013.

**Figure 9:** Isocontour surfaces for threshold value determination, in stress [17]. Images obtained in Radiation Physics Unit, University Aretaieio hospital, Athens, Greece, 2013.

**Figure 10:** 3D volume of a normal myocardium reconstruction is obtained through a specified MatLab code in order to compare the different filters used. Butterworth (a) and Hann (b) filetrs are used. Insignificant voxel differences are observed. Data acquired at Medical Imaging Nuclear Medicine and MatLab algorithm in Radiation Physics Unit, Aretaieion Hospital, Athens.

The article "Filters in 2D and 3D Cardiac SPECT Image Processing" was published in 2014. Journal: Cardiol Res Pract.

**Figure 11:** 3D myocardium processed by a MatLab code in order to compare myocardium volume at rest (left) and at stress (right) (Lyra et al, 2010). The image does not depict the real volume but the voxelized one (the functional myocardium). Figure is obtained from citation [18].
